The article "Radiological Analysis of COVID-19 Using Computational Intelligence: A Broad Gauge Study" was published in 2022. Journal: J Healthc Eng.

# Radiological Analysis of COVID-19 Using Computational Intelligence: A Broad Gauge Study

**DOI:** 10.1155/2022/5998042

**Published:** 2022-02-23

**Authors:** S. Vineth Ligi, Soumya Snigdha Kundu, R. Kumar, R. Narayanamoorthi, Khin Wee Lai, Samiappan Dhanalakshmi

**Affiliations:** ^1^Department of Electronics and Communication Engineering, College of Engineering and Technology, Faculty of Engineering and Technology, SRM Institute of Science and Technology, SRM Nagar, Kattankulathur, Chengalpattu, Chennai, TN, India; ^2^Department of Computer Science Engineering, College of Engineering and Technology, Faculty of Engineering and Technology, SRM Institute of Science and Technology, SRM Nagar, Kattankulathur, Chengalpattu, Chennai, TN, India; ^3^Department of Electrical and Electronics Engineering, College of Engineering and Technology, Faculty of Engineering and Technology, SRM Institute of Science and Technology, SRM Nagar, Kattankulathur, Chengalpattu, Chennai, TN, India; ^4^Department of Biomedical Engineering, Faculty of Engineering, Universiti Malaya, Kuala Lumpur, Malaysia

## Abstract

Pulmonary medical image analysis using image processing and deep learning approaches has made remarkable achievements in the diagnosis, prognosis, and severity check of lung diseases. The epidemic of COVID-19 brought out by the novel coronavirus has triggered a critical need for artificial intelligence assistance in diagnosing and controlling the disease to reduce its effects on people and global economies. This study aimed at identifying the various COVID-19 medical imaging analysis models proposed by different researchers and featured their merits and demerits. It gives a detailed discussion on the existing COVID-19 detection methodologies (diagnosis, prognosis, and severity/risk detection) and the challenges encountered for the same. It also highlights the various preprocessing and post-processing methods involved to enhance the detection mechanism. This work also tries to bring out the different unexplored research areas that are available for medical image analysis and how the vast research done for COVID-19 can advance the field. Despite deep learning methods presenting high levels of efficiency, some limitations have been briefly described in the study. Hence, this review can help understand the utilization and pros and cons of deep learning in analyzing medical images.

## 1. Introduction

The pandemic brought forth by the coronavirus disease 2019 (COVID-19) not only sustains a devastating response on the well-being and health of the worldwide population but also demands a high rate of monitoring so that it does not extend on its destructive path. A vital aspect of the battle against COVID-19 is the efficient examination of the patients, which can help the infected receive quick treatment and immediate care. As of now, the customary screening process to identify COVID-19 is the reverse transcriptase-polymerase chain reaction (RT-PCR) test method. This test identifies the presence of SARS-CoV-2 ribonucleic acid (RNA) in respiratory specimen samples (obtained via a range of procedures such as the nasopharyngeal or oropharyngeal swabs) [1]. The RT-PCR test method, despite being effective, has a few shortcomings. It is time-consuming, complicated, and involves a lot of manual labor. All these concerns make it difficult to comb through the highly populated regions where millions have to be tested in a rapid norm. It is also seen that the test's sensitivity aspect is highly variable [2, 3]. Radiographic examination was opted as recourse to surmount the difficulties in RT-PCR testing. Chest radiographs (computed tomography (CT) and chest X-ray (CXR) imaging) are imaged and examined by radiologists (as depicted in Figure 1(a)) to find visible references in tandem to the infection.

Preliminary studies discovered that patients affected by COVID-19 infection have abnormalities in chest radiographic images, with a few proposing that radiographic evaluation could be implemented as the principal method for COVID-19 screening in highly populated epidemic areas [4, 5]. Among radiographs, the CXRs are preferred over CTs [6] as they support rapid triaging in parallel to viral testing while being readily accessible and available. It is also easy to target multiple regions due to its portability. The more outstanding image quality of CT has to be sacrificed to avail these merits. Although the radiographs generated can significantly improve the process, it requires some form of automation. Doctors can hasten the diagnostic procedure, but it still involves scads of manual labor from skilled radiologists, which is not a feasible solution to tackle the large number of COVID-19 patients. To overcome this constraint, there have been constant research attempts utilizing deep learning (DL) methods to find the abnormalities (as seen in Figure 1(b)) in radiographs [7].

Convolutional neural network (CNN) is the primary choice of neural network framework for any DL practitioner working with medical images [8] and radiographs [9] along with vision-based tasks in general such as classification [10], object detection [11], and segmentation [12]. DenseNet, a type of CNN that forms the base to many of the architecture used to recognize COVID-19 from CTs and CXRs, is shown in Figure 2. CNNs stem from the mathematical operation of convolutions (as shown in Figure 3), which expresses the shape modification of functions. The term convolution encompasses the process and its result function. The ability of CNNs to analyze and capture spatial information helps to perform better than most other algorithms present. CNNs generally comprise convolutional layers, pooling layers, and various filters. The architecture usage depends on the demand and size of data available with which it is training. Dropout [13] and transfer learning [14] are commonly used techniques to improve the model's performance. Normalization approaches such as batch normalization [15] and group normalization [16] help improve the model's performance, provide the ability to users in building larger models, and tackle the vanishing gradient problem.

Machine learning (ML) algorithms are generally chosen over DL algorithms to compensate the computational requirements, but in the medical field, time and computational requirements are always traded off for higher standards of precision and hence used in preprocessing [19], feature selection [20], classification [21], and regression [22]. As the COIVD-19 demanded faster results, machine learning avenues have been explored (as shown in Table 1) to account for the global situation constraints. The outline of the application of the COVID-19 detection system in the real world is pictorially represented in Figure 4. In [18], an extensive study comparing K-nearest neighbor (KNN) and support vector machine (SVM) to CNNs was made. The experimentation presented that the DL classifiers trump the machine learning classifiers. Additionally, the DL-based classification methods generate results nearly 5 times faster than the machine learning classifiers. Hence, they are applied in various fields [23–26]. On experimentation with MobileNetV2 [27], the run time and computational power requirements were further reduced.  Table 2 lists the history of the networks used.

A simple inference that can be made throughout all the literature is that the DL models (especially CNNs) surmount the ML models due to their capability of capturing spatial information. The spatial correlations are completely absent in general ML methods and hence fail to capture important correlations or key points that are absent while considering the image in a linear aspect. The DL models are ultimately black box models, and the ML methods are easily interpretable. Still, recent explainable methods such as class activation maps [48, 49] help remove that barrier and let the user know how the model is providing an output or how the inference is generally created [50, 51].

### 1.1. Review Outline

The following contributions are made through this review study:

- A detailed discussion is done with respect to the COVID-19 prediction approaches of the preceding reviews. The study analyses their merits and demerits and provides key insights as well regarding the same. It covers the essential aspects of COVID-19 research that the previous studies have missed.
- A systematic comparison is studied encompassing COVID-19 detection techniques about prognosis, diagnosis, and severity/risk detection.
- An extensive discussion on the challenges with regard to fostering high-quality results in detecting COVID-19. Solutions for these challenges are presented alongside as well.
- An in-depth analysis of the pre- and post-processing methods used on the COVID-19 datasets and architectures is provided.
- Discussion on the unexplored areas such as meta-learning and self-supervised learning and defining the explorable research avenues regarding the same are presented.
- This work emphasizes how most of the research that takes place for COVID-19 can help propagate research for other diseases and medical image analysis in general.

Moving on to Section 2, the discussion is carried out regarding the premier approaches in COVID-19 detection methodologies on diagnosis, prognosis, and severity/risk detection. The inferences collected from reviewing the papers are also noted.  Section 3 discusses the merits and limitations of the past reviews, which have described past attempts on detecting COVID-19 through deep learning methods. The section also includes an extension to the solutions provided to the challenges mentioned in Shorten et al. [52] by exploring different paradigms of deep learning. A discussion on the various vision-based pre- and post-processing techniques used to improve deep learning algorithms is given in Section 4. The review continues by identifying more challenges faced while attempting to detect COVID-19 and a brief discourse on the future directions to utilize the vast research done for COVID-19 towards the domain of medical image analysis in general under Section 5 and the conclusion in Section 6.

## 2. Discussion on COVID-19 Medical Image Analysis

The major COVID-19 medical image analysis tasks are as follows: diagnosis, prognosis, and severity/risk detection. The upsurge of the COVID-19 epidemic has triggered many researchers to contribute their research findings in pulmonary image analysis using DL and other image processing techniques leading to an astonishing breakthrough in COVID-19 diagnosis with stupendous amount of quality works. Discerning COVID-19 from other non-COVID-19 conditions is an important issue to be addressed; hence, the study has been majorly categorized as follows: COVID-19/non-COVID-19 pneumonia (2-class classification) and COVID-19/non-COVID-19 pneumonia/normal (3-class classification). The study also includes a discussion on classifying COVID-19 against normal condition and other lung diseases, the impact of 2-class and 3-class classifications using the same algorithm on the same dataset, and performing the same classification technique on different image modalities (CT and CXR). The aforementioned workflow has been pictorially depicted in Figure 5.

### 2.1. COVID-19 Diagnosis

COVID-19 diagnostic approach based on medical image analysis utilizes the CXR and CT images. AI can adequately improve the diagnostic model's efficiency by accurately locating the infections due to the virus in X-ray and CT images, hence facilitating assistance to the radiologists in making clinical decisions for disease diagnosis and triage. [53].

#### 2.1.1. COVID-19/Non-COVID-19 Pneumonia Diagnosis

Harmon et al. [54] proposed an AI-based 3D model using DenseNet-121 to identify COVID-19 from multinational CT data. 2724 scans from 2617 COVID-19 victims were used in this work, among which 1029 scans belonged to 922 RT-PCR-confirmed COVID-19 patients. Initially, the lung region was segmented using Anisotropic Hybrid-Net (AH-Net) architecture. On testing the model using an independent dataset, it achieved accuracy of 90.8%, area under the curve (AUC) of 0.949, sensitivity of 84%, specificity of 93%, positive predictive value (PPV) of 0.794, and negative predictive value (NPV) of 0.984 with sufficient generalization. In 140 non-COVID-19 pneumonia patients, the false-positive rate was 10%. This model was able to furnish reasonable performance metrics, thereby enabling it as an unbiased clinical trial tool for assisting the COVID-19 medical image analysis in specific bounded societies during the epidemic outbreak.

A dual-sampling attention network realized by a 3D CNN using ResNet-34 with an online attention refinement and a dual-sampling strategy was proposed by Ouyang et al. [55] to categorize COVID-19 against community-acquired pneumonia (CAP). The model was evaluated on a multicenter CT dataset of 4982 images consisting of 1593 CAP and 3389 COVID-19 images. Dual-sampling strategy (uniform sampling and size-balanced sampling) was used to mitigate the effect of imbalanced learning and the online attention module to target the infected regions, thereby increasing the model explainability and interpretability by showing visual evidence to reveal the critical regions considered by the model for diagnosis. The ability to generalize the proposed model was evaluated using an autonomous test data, which gave an accuracy of 87.5%, AUC value of 0.944, along with sensitivity of 86.9%, specificity of 90.1%, and *F*1 score of 82.0%.

A multiview fusion model using ResNet-50 was developed by Wu et al. [56], which makes use of the axial, sagittal, and coronal views of CT as the three-channel input image to the model. A multicenter dataset consisting of high-resolution CT images of 368 COVID-19-infected patients and 127 patients suffering from other pneumonia (67 viral pneumonia, 47 bacterial pneumonia, 11 mycoplasma pneumonia, and 2 fungal pneumonia) were collected. The multiview model shows better performance than the single-view model with an accuracy of 76%, AUC value of 0.819, sensitivity of 81.1%, specificity of 61.5%, and overcoming the overfitting issue of the single-view model. This model can mitigate the work burden of radiologists and hence improve the diagnostic efficiency.

Ardakani et al. [57] compared ten convolutional neural networks: ResNet-101, ResNet-50, ResNet-18, VGG-16, VGG-19, MobileNetV2, SqueezeNet, AlexNet, GoogLeNet, and Xception to distinguish COVID-19 against non-COVID-19 pneumonia. A dataset consisting of 1020 high-resolution CT scan slices from 108 COIVD-19 victims and 86 victims with non-COVID-19 pneumonia (viral pneumonia and other atypical pneumonia) were collected. ResNet-101 surpassed the other CNNs due to its high sensitivity of 100% and AUC value of 0.994 for the given dataset. It also achieved accuracy of 99.51%, specificity of 99.02%, PPV of 99.03%, and NPV of 100%. This model is claimed to remove the substantial cost and can be used as an ancillary method in CT imaging.

An adaptive feature selection-guided deep forest (AFS-DF) method was proposed by Sun et al. [58] for COVID-19 classification using CT radiographs. The deep forest model was used on four location-specific handcrafted features such as volume, surface area, number of infected lesions, and histogram distribution from the CT images to describe high-level feature representation. The selected features were classified using SVM. A dataset consisting of 2522 de-identified pulmonary CT images from 1027 CAP and 1495 COVID-19-infected patients was used for this study. The proposed AFS-DF variants outperform by achieving 1.38%, 1.15%, and 1.11% enhancement over their obverse methods (logistic regression (LR), SVM, and RF) in most of the evaluation metrics. AFS-DF-SVM outperforms the other models with accuracy of 91.79%, AUC value of 0.9635, sensitivity of 93.05%, and specificity of 89.95%. ASF-DF reduces the repetition of features using the trained forest.

In the study by Narin et al. [59], binary classifications were performed to distinguish COVID-19 against viral and bacterial pneumonia using 341 COVID-19 CXRs and 2800 normal CXRs from the GitHub repository (open source) commonly contributed by Cohen et al. [60] and ChestX-ray8 database [61], respectively. 2772 bacterial pneumonia and 1493 viral pneumonia CXRs were collected from a Kaggle repository called chest X-ray images (pneumonia) [62]. The model performance of five different pre-trained CNN variants (ResNet-152, ResNet-101, ResNet-50, Inception-ResNetV2, and InceptionV3) was compared, among which ResNet-50 model showcased the highest classification performance. This model achieved an accuracy, precision, and specificity of 99.5%, 98.0%, and 99.5%, respectively, for discriminating COVID-19 against other viral pneumonia, whereas for COVID-19/bacterial pneumonia classification, the accuracy, precision, and specificity values were 99.7%, 98.3%, and 99.8%, respectively. This method was implemented directly in an end-to-end manner eliminating manual intervention for feature extraction, feature selection, or classification tasks.

A deep learning model comprising of three major components, a backbone network, a classification head, and an anomaly detection head, was proposed by Zhang et al. [63] to reduce the false-negative rate as much as possible. The model was built using 1431 CXR pneumonia images of 1008 patients from the ChestX-ray14 dataset [61] and 100 images belonging to 70 COVID-19 patients from the GitHub repository [60]. The experiment was conducted for different values of *T* parameter that controls the compensation between the true-positive rate and the true-negative rate. As the *T* value decreases from 0.50 to 0.15, the sensitivity increases from 72.00% to 96.00% and the specificity drops from 97.97% to 70.65%, but the AUC value remains the same. Based on the performance metrics (sensitivity—96%, specificity—70.65%, and AUC—95.18), the model performs well for *T* = 0.15 with a reduced false-negative rate of nearly 4%. Despite its good performance, it had its limitations, 4% missing COVID-19 cases and a false-positive rate of almost 30%.

Abraham and Nair [64] used a combination of multi-CNN models (MobileNetV2, SqueezeNet, Xception, DarkNet-53, and ShuffleNet) with correlation-based feature selection (CFS) followed by the BayesNet classifier. The experiment was performed using two datasets: Dataset I: 453 COVID-19 and 107 non-COVID-19 images of either bacterial/viral pneumonia [55] and 390 CXRs of viral and bacterial pneumonia [60, 61, 65, 66] and Dataset II: 71 COVID-19 CXRs and 7 non-COVID-19 CXRs [66]. Only the BayesNet classifier achieved an accuracy of >90%. The proposed model gave an accuracy of 91.16% and 91.44% for Dataset I and Dataset II, respectively. The multi-CNNs (with 3 or more pre-trained CNNs) comparatively showed better results than the single pre-trained CNNs.

Autee et al. [67] proposed the StackNet-DenVIS to reduce the false-negative rate in classification using a stacked generalization ensemble of four different CNNs. A total of 9953 CXRs consisting of 9085 non-COVID-19 and 868 COVID-19 cases from multiple sources were gathered [60, 65, 68, 69]. The data imbalance problem was handled by generating synthetic images using deep convolutional adversarial generative networks and SMOTE + Tomex links. With an accuracy of 95.07%, this model achieved a low false-negative rate at low cost in comparison with the RT-PCR test.

#### 2.1.2. COVID-19/Non-COVID-19 Pneumonia/Normal or Non-Pneumonia Diagnosis

A 3D deep learning framework, COVNet, realized using ResNet-50 was implemented by Li et al. [70] to distinguish COVID-19 against CAP and non-pneumonia cases. The network was able to extract the 2D local features and the 3D global representative features for better classification. A CT image dataset consisting of 1292 COVID-19 CTs, 1325 CTs with non-COVID-19 pneumonia, and 1735 CTs with CAP infections, totally contributing to 4352 scans, was collected for this study. An AUC value of 0.96, sensitivity of 90%, and specificity of 96% were obtained with 95% confidence interval for an independent test dataset. Due to the shortage of laboratory-confirmed COVID-19 data, the work was unable to present the results for distinguishing COVID-19 from other lung diseases.

Wang et al. [71] have proposed a prior-attention residual model, PA-66-M, using two subnetworks based on 3D ResNets for pneumonia detection and classification of pneumonia type. The two subnetworks were integrated by a late-fusion strategy using a fully connected layer with learning capacity. Lung segmentation was performed using U-Net. The dataset consisting of 936 chest CTs of normal cases, 2406 CT images with interstitial lung disease (only viral pneumonia), and 1315 COVID-19-infected CT images was collected from multiple cooperative hospitals. The proposed model was capable of accurately focusing the lesions with an accuracy, sensitivity, and specificity of 93.3%, 87.6%, and 95.5%, respectively. By applying a constant weighting factor, the prior-attention residual model was able to converge faster than the self-attention strategy. Some of the normal scans were misclassified to pneumonia class by the proposed model, and it also failed to unveil some of the scans with COVID-19 lesions.

Hasan et al. [72] used handcrafted texture features based on Q-deformed entropy along with deep features from CNN. The extracted features were refined by analysis of variance (ANOVA) and then classified to distinguish COVID-19 from other pneumonia types and normal cases. The LSTM neural network classifier outperformed SVM, KNN, and LR with an accuracy of 99.68%. The performance of the combined features was better when compared to using only handcrafted or deep features.

Three-dimensional classification models using two CNNs namely the ResNet-23 and ResNet-18 were used by Butt et al. [73] to classify COVID-19/influenza A viral pneumonia (IAVP)/normal CT image patches. A location attention mechanism was incorporated to identify the corresponding location of the identified patch in the pulmonary CT image. This model was smart enough to accurately distinguish COVID-19, when compared to using a model without location attention mechanism. Hence, an overall accuracy of 86.7% was observed with sensitivity of 98.2%, specificity of 92.2%, and AUC value of 0.996. This work used 618 transverse-section CT samples in which 219 samples were obtained from nearly 110 COVID-19-infected patients, 224 scans from 224 IAVP patients, and 175 from healthy people.

Detailed relation extraction neural network (DRENet) is a pre-trained ResNet-50 with feature pyramid network proposed by Song et al. [74] to derive the top-K-level features and extract the image-level predictions for COVID-19 diagnosis at the patient level. For model development and evaluation, the dataset was collected from different hospitals comprising 777 CT images from 88 COVID-19 victims, 505 CT slices from 100 bacterial pneumonia patients, and 708 CT slices from 86 healthy people. The regions detected by the proposed model contained the most important feature of COVID-19 infection, ground-glass opacity (GGO). DRENet exhibited an efficient performance with an accuracy of 93% and F1 score of 0.93.

A social mimic optimization method was proposed by Toğaçar et al. [75] to select the potential deep features from the combined feature set of MobileNetV2 and SqueezeNet, to categorize COVID-19 from pneumonia and normal conditions. It provides efficient features by stacking the original images with the reconstructed fuzzy color images, which had better quality and reduced noise. It used 76 COVID-19 images from [60] and 295 COVID-19, 98 pneumonia, and 65 normal images from [69]. On classification using SVM, all performance metrics, F score, sensitivity, specificity, precision, and accuracy, were 100% for detecting COVID-19 cases, exhibiting an overall accuracy of 99.27%. The average values of F score, sensitivity, specificity, and precision for all the three classes are 0.9858, 98.33%, 99.69%, and 98.89%, respectively. The model was aimed to produce swift and more authentic results as MobileNetV2 and SqueezeNet used fewer parameters compared with the other networks.

Wang et al. [68] created an open-source network, COVID-Net, and public dataset, COVIDx, consisting of 13,975 CXR images belonging to 13,870 patients obtained by combining data from five different public data repositories [60, 76–79]. COVID-Net architecture used a lightweight residual design pattern called projection-expansion-projection-extension (PEPX) pre-trained on ImageNet dataset.

Compared with VGG-19 and ResNet-50 architectures, COVID-Net has lower complexity in terms of architecture and computations. It showed an accuracy of 93.3% with sensitivity of 91.0%. Qualitative analysis of the network implies that it does not depend on inappropriate information for decision-making.

Nishio et al. [80] have evaluated the performance of conventional neural network architectures with different data augmentation techniques (conventional method, mix up, and random image cropping and patching (RICAP)) to identify COVID-19 pneumonia from pulmonary X-rays. 215 COVID-19-infected, 533 non-COVID-19 pneumonia-infected, and 500 healthy CXR images [60, 80] were used for this work. VGG-16 with the combination of conventional with mix-up data augmentation was found to give better results with an accuracy of 83.7% and a sensitivity value of 90.9% compared with ResNet-50, DenseNet-121, MobileNet, and EfficientNet.

The MH-Net proposed by Canayaz et al. [81] makes use of two meta-heuristic algorithms namely the binary gray wolf optimization (BGWO) and binary particle swarm optimization (BPSO) to select the potential features extracted from VGG-19, ResNet, GoogLeNet, and AlexNet. Finally, an SVM classifier was used. 364 CXR images each of COVID-19, pneumonia, and normal cases ([60, 65, 69]) enhanced by the image contrast enhancement algorithm were used for this work. VGG-19 model with BPSO feature optimization (488 features) on the enhanced data outperforms the other models with an overall accuracy of 99.38%, sensitivity of 99.39%, and specificity of 99.69%. The unbalanced class problem is overcome using equal number of CXRs in each class, and also, it uses fewer parameters compared with other models.

The COVID-19 Inception-ResNet model (CoVIRNet) that uses different inception residual blocks for diagnosing COVID-19 infection from the CXR images was proposed by Almalki et al. [82]. Multiscale feature maps obtained from different depths, which are then concatenated by average pooling, are used to improve the efficiency of the proposed method. The problem of overfitting encountered by small datasets has been overcome using different regularization techniques in the deep learning blocks. The author proposed two approaches: (i) CoVIRNet-Inception-ResNet blocks consisting of a single inception module with extra branches of convolution layer using reduction factorization; (ii) CoVIRNet with RF-multiscale, multilayer features extracted from the proposed Inception-ResNet blocks are classified using a random forest classifier. For this, a multicenter dataset of size of 1251 was used, among which 284 COVID-19 infection images were collected from [79, 83]. 310 normal CXRs, 330 bacterial pneumonia, and 327 viral pneumonia-infected images were collected from [62]. On comparing the performance of CoVIRNet with fine-tuned versions of Xception, ResNet-101, MobileNetV2, and DenseNet-201, the second approach CoVIRNet with RF showed better performance with accuracy of 97.29%, precision of 97.74%, recall of 97.02%, and *F* score of 0.9732.

Subsection 2.1 gives a brief review on the different COVID-19 diagnostic methods by performing two-class or three-class classifications against other pneumonia/normal cases proposed by various researchers in both CXR and CT imaging modalities. Tables 3 and 4 summarize the studies including the network, dataset, and performance metrics used for the evaluation of COVID-19/non-COVID-19 pneumonia diagnosis and COVID-19/non-COVID-19 pneumonia/normal or non-pneumonia diagnosis, respectively. The performance metrics used for evaluation and their corresponding formulae are tabulated in Table 5.

#### 2.1.3. Other Comparative Studies

Apart from the techniques mentioned in the previous sections, there are also other comparative studies done by some researchers, which explore the performance of a COVID-19 diagnostic algorithm for different image modalities (CT and CXR) or on datasets with binary (COVID-19/non-COVID-19) or multiclass classifications (COVID-19/non-COVID-19/normal/other lung diseases).

*(1) Comparison of Binary and Multiclass Classification*. Hu et al. [84] performed an automated diagnosis of COIVD-19 based on ShuffleNetV2 on pulmonary CT images. Two classifications are performed on the data collected from multiple sources. 16 different data augmentation operations were performed on the 1042 chest CT images (comprising of 521 COVID-19, 397 healthy, 76 bacterial pneumonia, and 48 SARS) to increase the dataset size for better training of the model. Binary classification of COVID-19 from the healthy cases obtained an accuracy of 91.21% along with sensitivity of 90.52%, specificity of 91.58%, and AUC value of 0.9689. In the case of multiclass classification (COVID-19/bacterial pneumonia/SARS), the accuracy dropped to 85.40% for the same algorithm. The sensitivity, specificity, and AUC values were 85.71%, 84.88%, and 0.9222, respectively.

Chowdhury et al. [69] had compared the performance of different pre-trained CNNs for COVID-19 detection with and without data augmentation using the data collected from multiple public datasets ([60, 83, 85]). Among the various networks analyzed, DenseNet-201 showed comparably better classification results for both COVID-19/normal and COVID-19/normal/pneumonia discrimination with image augmentation. The binary classification shows better performance with an accuracy of 99.7% compared with the multiclass problem with an accuracy of 97.94%. The performance difference was insignificant, and the overall performance of three-class problem was less in comparison with the binary classification problem.

COVID-DenseNet proposed by Sarker et al. [86] is a deep learning architecture realized using DenseNet-121 with transfer learning from CheXNet for the detection of COVID-19 from COVIDx [71] CXR images. The most significant regions in the image that were responsible for the prediction were highlighted by performing an interpretation analysis using Grad-CAM. The overall accuracy for COVID-19/non-COVID-19 classification and COVID-19/pneumonia/normal classification is 0.96 and 0.94, respectively. This work tried to make the model explainable and interpretable to certain extent using the Grad-CAM representation.

DarkCovidNet architecture based on the DarkNet-19 model was designed by Ozturk et al. [87] to identify COVID-19 from X-ray images collected from [60, 61] comprising of 127 COVID-19, 500 pneumonia, and 500 normal images. For COVID-19/no findings/pneumonia classification, the model produced a classification accuracy, sensitivity, and specificity of 87.02%, 85.35%, and 92.18%, respectively. In the case of binary classification COVID-19/no findings, the performance metrics increased to accuracy of 98.08%, sensitivity of 95.13%, and specificity of 95.3%. DarkCovidNet was able to diagnose COVID-19 within seconds.

Mahmud et al. [88] proposed the CovXNet architecture, which is a multi-dilation CNN architecture that makes use of transferable multi-receptive feature optimization technique for COVID-19 detection from CXR images. A balanced dataset consisting of 305 images of different resolutions collected from different medical centers was used for each class: COVID-19, viral pneumonia, bacterial pneumonia, and normal. For distinguishing COVID-19 against normal, bacterial pneumonia, and viral pneumonia, the binary classification resulted in a accuracy of 97.4%, 94.7%, and 87.3%, respectively. While carrying over the same architecture for multiclass classifications such as COVID-19/viral pneumonia/bacterial pneumonia and COVID-19/normal/viral pneumonia/bacterial pneumonia, the classification accuracies dropped to 89.6% and 90.2%, respectively. Based on the obtained results, distinguishing viral pneumonia from COVID-19 is arduous when compared to other diseases. CovXNet is highly scalable with huge receptive capacity.

*(2) Comparison of COVID-19 Diagnostic Performance in CT and CXR Images*. COVID-MTNet is a deep learning architecture proposed by Alom et al. [89] to perform multiple tasks such as COVID-19 segmentation and detection from CT and CXR images. A dataset of 3875 samples of COVID-19 pneumonia and 1341samples for normal cases was collected from [60, 62]. The infected regions were segmented using the NABLA-N network, and the detection process was performed using the inception recurrent residual neural network (IRRCNN) model with transfer learning. The segmentation network using pixel-level analysis significantly reduced the possibility of false-positive and false-negative detections. The model produced a segmentation accuracy of 94.52% for CXR images and 99.56% for CT images in the test data. In the detection model, an accuracy of 98.78% and 87.26% was observed in the CT and CXR images, respectively. These results show that the CT imaging modality better discriminates the COVID-19 infection from the normal cases. The detection model can be generalized and made to produce more accurate results by training greater number of samples. Some false-positive detections were observed in the segmentation model for CT images due to the insufficiency of labeled CT data for COVID-19 infection.

Vinod and Prabaharan [90] proposed an artificial intelligence technique for fast COIVD-19 diagnosis using decision tree classifier with deep CNN features. The CXR dataset contains 113 normal images and 306 COVID-19-infected X-rays. The CT dataset contains 350 COVID-19 images and 395 non-COVID-19 images. The test score resulted in 0.82 for CT and 0.87 for CXR. The recall score is high in the case of CT images, i.e., 0.93. The recall score for COVID-19 diagnosis in CXR images is 0.88. The number of false negatives is less for diagnosis in CT image modalities.

In [91] by Perumal et al., Haralick texture features were extracted from the enhanced images. These modified images were then fed into different predefined CNN models such as ResNet-50, VGG-16, and InceptionV3 to find the patterns similar to other pneumonia, so that it can easily detect COVID-19 across other diseases. 14 Haralick features (mean, variance, entropy, etc.) were used for the identification of the relationship between biological features in the data. This method was experimented on data from multiple centers ([60, 65, 92, 93]). VGG-16 using transfer learning achieves better classification with an accuracy of 93%, precision of 91%, and recall of 90%.

Irfan et al. [94] developed a hybrid multimodel deep neural network (HDNN) for COVID-19 detection from multimodal data. It was designed as a mixture of LSTM and CNN to predict the risk of disease onset from both CT and CXRs. 1500 images from healthy patients and 3500 images from infected (COVID-19 and pneumonia) patients were collected from various sources ([60, 77, 78, 95, 96]). Initial preprocessing involves the Kalman discrete-time model-based denoising followed by sampling the 1080 × 1080 sized images to 256 × 64 sized time-series data. The hybrid model added efficacy to the work using LSTM to vanish the gradient problem and CNN to extract features automatically. On classifying the data into normal, pneumonia, and COVID-19-infected, an accuracy of 99% and PPV of 98.7% were obtained. This work also concludes that COVID-19 detection from CTs using HDNNs proves to be consistent and fast.

Other approaches that include classification of COVID-19-positive cases against COVID-19-negative cases or healthy cases [97–99] were present and also classification of COVID-19 against other pulmonary diseases as in [100], where a deep neural network with the generative adversarial network (GAN) based on synthetic data augmentation is used to classify 8 different lung pathologies. The collected dataset contains images from Digital Pathology Classification Challenge (Kaggle) and COVID-19 images from [60] comprising of 5789 atelectasis, 1010 cardiomegaly, 6331 effusion, 10317 infiltration, 6046 mass, 1971 nodule, 1062 pneumonia, 2793 pneumothorax, 84312 normal, and 337 COVID-19 images. The proposed model performed better than InceptionV3 and ResNet models with an accuracy of 89.2%. Accurate lung region of interest (ROI) segmentation also takes an indispensable part in better diagnosis of COVID-19 by delineating the lesions and measuring their extent. Most of the works have used U-Net [101] architecture for this purpose ([70, 71, 95, 102]). U-Net is a CNN architecture developed specially for biomedical image segmentation with the ability to give both the localization information and the contextual information, which leads to the better prediction of a segmentation map. Image segmentation can also be applied to quantify the lung-infected region ([101, 103, 104]), which involves visualization of the lesion distribution, prediction of severity, and assessing the progression during follow-up.

### 2.2. COVID-19 Prognosis

Prognosis refers to predicting the likeliness or expected disease development based on the track of the disease that is diagnosed, the condition of the patient (physical and mental), the available treatments, and other additional factors. Few COVID-19 prognosis methods are explained in this section.

Sverzellati et al. [105] simulated the triage setting of a pandemic environment with large population of COVID-19-infected suspects provided that the clinical decision should be given in the absence of any resource constraints. For this, reconstructed CXR (r-CXR) images were generated from the high-resolution CT (HRCT) images. Mortality prediction was done based on the multivariable (age, sex, duration of symptoms at triage, and a comorbidity score of 0–4) by performing LR analyses to identify the contribution of clinical and radiological variables in the analysis and using a study population of 300 patients. The images were graded as follows: normal, alternative diagnosis (to be specified), indeterminate, or typical for COVID-19 pneumonia by expert radiologists. The study findings put forward that the clinicians can rely on positive CXR for showing the low or high extent of pneumonia, and in the case of the intermediate extent of CXR, it is complemented by CT for optimal stratification of high- and low-risk groups. For indicating the COVID-19 infection, the sensitivity, specificity, PPV, and NPV of HRCT are 95.2%, 32.8%, 82.2%, and 67.9%, respectively, which proves to be better than the corresponding metrics of r-CXR.

Wang et al. [106] proposed the COVID-19Net to identify patients of potentially high risk with poor prognosis using the transfer learning process in two steps. Initially, the network was trained on 4106 non-COVID-19 CT images from epidermal growth factor receptor (EGFR) dataset, which was then transferred to the COVID-19 dataset consisting of CT images from 1266 victims: 924 with COVID-19 (471 patients had follow-up for more than 5 days) and 342 with other pneumonia. For prognostic analysis, 64-dimensional DL features were combined with clinical features (age, sex, and comorbidity) to compose an integrated feature vector. Then, a multivariate Cox proportional hazard model was used to predict the risk of a patient. The Kaplan–Meier analysis and log-rank test implied that the deep features have promising prognostic value for COVID-19 (*p* < 0.0001, *p*=0.013, and *p*=0.014 in 3 datasets).

Feng et al. in [107] explored the predictive value of COVID-19 prognosis from chest CT images by comparing the difference in clinical and CT characteristics in the progressive and stable patients by performing multivariate LR and nomogram establishment. Older age, CT severity score on admission, and higher neutrophil-to-lymphocyte ratio (NLR) were identified to be the independent and significant predictive aspects for advancement to severe COVID-19 infection during hospitalization and were supported by an appreciative calibration of the nomogram, a nonsignificant Hosmer–Lemeshow test statistic (*p*=0.791), and AUC value of 0.898 in the validation cohort. This method was simple with only three easily obtainable variables and was capable of promptly predicting the progression risk (in-hospital) in the moderate stage of COVID-19 patients within 14 days. It was performed on an unbalanced data consisting of only 10% of patients developing severe COVID-19 pneumonia, which seems to be a limitation of this work.

Liang et al. [108] developed and validated a risk prediction method for early diagnosis of COVID-19 infection in patients. For this, different clinical, laboratory, epidemiological, and radiological image variables were screened at the time of admission in medical center/hospital to predict the risk score as low-, moderate-, and high-risk cases. The Least Absolute Shrinkage and Selection Operator (LASSO) was used for screening the variables, and LR was used to formulate the predictive risk score (COVID-GRAM). This method was developed with a cohort of 1590 patients and validated on 710 patients to estimate the risk that they will develop a critical illness. 10 variables including chest radiographic abnormality, age, cancer history, number of comorbidities, and NLR were identified as independent predictive factors among 72 potential factors by the LR model. A mean accuracy of 0.88 was obtained in the validation group. This was designed as a Web-based calculator to assist the clinicians in estimating the possibility of developing critical ailment in individual hospitalized victims. As the development and validation patient group was completely selected from a particular county, there might be limitation in generalizing the work for patients from different regions.

Wu et al. [109] used CT images to develop an easy-to-use and noninvasive prognosis method to predict the clinical risk of COVID-19 patient outcome as death, need for mechanical ventilation, and admission to the intensive care unit. The development cohort consists of 492 patients grouped into the early-phase group and the late-phase group based on their CT scanning performed one week before or after the symptom onset, respectively. A fine-gray competing risk regression model was used to frame the clinical model and CrrScore (the clinic-radiomic signature), and a Least Absolute Shrinkage and Selection Operator (LASSO) was used to construct the RadScore (the radiomic signature). In the late-phase group, the radiomic signature alone proved to be efficient to forecast the poor outcome in patients with an AUC value of 0.976 and C-index of 0.885. In the case of the early-phase group, the clinic-radiomic signature exhibited better efficacy with an AUC value of 0.862 and C-index of 0.850. Therefore, based on the time of CT scanning concerning the symptom onset, appropriate signatures can be used for predicting the prognostic outcome.

Research works on the prognostic analysis of COVID-19 using radiological images are minimal and need to be further explored to keep a check on the severity of the diseases and reduce the mortality rate. For prognosis, the clinical features are combined with the radiological image findings to predict the patient's medical condition for delivering successful triage and lessen the disease spread.

### 2.3. COVID-19 Severity/Risk Detection

A streamlined severity/risk detection mechanism is highly required for COVID-19 triage to lower the prodigious rate of mortality. Apart from early screening, the severity assessment also plays a vital role in triage and disease management. A review on the related works in the literature is discussed below.

Cohen et al. [110] built a severity prediction model to assist the clinicians in managing the patient care using a regression model to predict two types of scores: extent of lung involvement (0–8 score) by ground-glass opacity or consolidation and degree of opacity (0–6 score) on the COVID-19-infected CXR images. DenseNet was employed to predict pneumonia from 94 COVID-19 CXR images acquired from [8]. The model was trained with 7 datasets [90, 98, 111–115] with 18 common radiological finding tasks consisting of 88,079 non-COVID-19 CXR images. Just using a single feature (lung opacity) for risk predictions countered to the ground truth value of prediction score, the model was capable of better prediction in both the opacity score and the geographic extent of infection. The Pearson correlation coefficient and *R*^2^ for lung opacity score prediction task are 0.78 ± 0.04 and 0.58 ± 0.09, respectively. Similarly, for the geographic extent prediction the Pearson correlation coefficient of 0.80 ± 0.05 and *R*^2^ value of 0.60 ± 0.09 were obtained. It was capable of predicting the geographic extent score (range 0–8) with 1.14 mean absolute error (MAE) and lung opacity score (range 0–6) with 0.78 MAE generalization that can be improved by performing large-scale evaluations on public datasets from around the world.

Zhu et al. [116] also employed a model similar to [110] for accurate staging of COVID-19 severity on CXRs. A deep CNN model was used to foresee the lung severity scores from 131 CXRs based on the degree of opacity (0–3 score) and geographic extent (0–4 score). A correlation analysis was performed amidst the predicted score and the radiologist scores, which resulted in a higher value of 0.90 and a MAE of 8.5%, making the model yield top results. An average opacity score of 2.52 and average geographic extent score of 3.42 were obtained across three readers.

Tang et al. [17] proposed a severity assessment model to categorize the COVID-19-infected CT images as severe or non-severe. For these, 63 quantitative features of top importance such as volume and ratio of the left/right/whole lung and volume of GGO were extracted from 176 CT images obtained from different hospitals (using different scanners) and trained to the random forest model. An accuracy of 0.85, AUC value of 0.91, true positive rate of 0.933, and true negative rate of 0.745 were obtained for this model. The volume and ratio of GGO were identified to be the feature with most importance to estimate the severity of the disease, and another finding from the study revealed that the quantitative features observed in the right lung were more significantly related to COVID-19 severity than the features of the left lung. The main drawback is that the model is able to label the images as only severe or non-severe instead of multiple classifications such as mild, common, severe, and critical.

The limitation of [17] can be overcome by the COVID-SDNet proposed by Tabik et al. [117], which has better generalization capability. A balanced and homogeneous database, COVIDGR-1.0, was built, which includes different levels of severity such as normal with positive RT-PCR (normal PCR+), mild, moderate, and severe. It consists of 426 COVID-19-positive CXR images and 426 COVID-19-negative images (normal PCR: 76, mild: 100, moderate: 171, and severe: 79). It performs smart data generation using a class-inherent transformation approach motivated by GAN and ResNet-50 loaded with ImageNet weights for classification. Better and more stable results and great balance between specificity and sensitivity were obtained. Comparing the classification accuracies of 4-class classification (normal PCR +: 28.42% ± 2.58, mild: 61.80% ± 5.49, moderate: 86.90% ± 3.20, and severe: 97.72% ± 0.95) and 3-class classification (mild: 46.00% ± 7.10, moderate: 85.38% ± 1.85, and severe: 97.22% ± 1.86), even though normal PCR + seems to be the toughest level to predict, its existence accelerates the accuracy of the minor severity levels, notably mild level. It is also observed that the segmentation of the lung region using U-Net has essentially improved the sensitivity value.

Severity assessment in COVID-19 mostly relies on classifying the pre-identified radiological images or using the clinical data of patients to perform the severity analysis, but pre-identification of radiological images as mild, moderate, or severe infections may be challenging and difficult.

### 2.4. Inferences

Based on the study described in the previous sections, the review findings and inferences are listed below:

- COVID-19 diagnosis can be performed by classification or segmenting the infected region. Classification can be viable and easy to implement in short time as it demands only weak image-level labels and few model specifications for training the classification model.
- Classification of COVID-19 infection against normal cases seems to be much easier with high classification results and performance metrics. In general, binary classification (COVID-19/non-COVID-19, COVID-19/other pneumonia) yields better results than multiclass classification (COVID-19/other pneumonia/normal/other lung diseases).
- Distinguishing COVID-19 from other pneumonia, especially viral pneumonia, is challenging as they show similar characteristics in the radiological images. In such cases, the efficiency of the classifier can be improved by adding more images or other types so that the learning process can be enhanced during training. The performance of distinguishing COVID-19 from normal or bacterial pneumonia can yield better results since there is significant variation in the radiological image features.
- Deep Learning methods are mostly preferred than the machine learning methods for feature extraction as they can extract the inherent deep features specific to each class for a finer classification. The most commonly used deep models for feature extraction and classification that give promising results are DenseNet, ResNet, VGG, and their modified variants. Other networks like Inception, Exception, ShuffleNet, and EfficientNet also have been used in many works. The CNN layer implementation with residual connection is depicted in Figure 6. Diagnosis of COVID-19 employing deep learning techniques have shown better sensitivity and specificity than the radiologist's decision. U-Net is the most widely preferred deep learning architecture for segmentation task, which is depicted in Figure 7.
- Deep features can be combined with clinical data such as clinical symptoms, nucleic acid detection results, epidemiology, and laboratory indicators, which can bypass any misdiagnosis and efficaciously improve the clinical triage.
- Prognosis of COVID-19 is of equal importance as that of diagnosis, since it demands medical triage and management of the patient care. Early identification of the disease can aid in the diagnostic ambiguity of radiologists. Works on COVID-19 prognosis are minimal, so this can open up a large research path for many researchers.
- Prediction of COVID-19 infection severity plays a vital role in making clinical decisions so that the medical team can work towards reducing the mortality rate.
- Despite CXRs being cheap and easily obtainable, CTs are highly preferred for COVID-19 analysis as they are capable of early detection of the disease even in victims with negative RT-PCR tests, in asymptotic patients or even ahead symptoms may arise.

Figure 8 illustrates the inferences from the review of different tasks related to medical image analysis of COVID-19.

## 3. Related Reviews in the Field

There are have been previous reviews [52, 118] that have encompassed most of the research regarding COVID-19 in terms of machine learning, deep learning, and medical imaging along with its analysis and scrutinized them to preference inferences, to promote further research in the field. They also present challenges that future researchers should tackle to incorporate better results and build more efficient models.  Table 6 (while there are other reviews present, they were either extremely short, or did not contain valuable information, or were mostly covered in the mentioned reviews.) lists out the most useful reviews, which have taken place till date and their respective merits and limitations. Most reviews covered the architectures used quite broadly and have also made studies in context to their usage (pre-trained or incorporation for custom methods). A general pipeline of the same is shown in Figure 9. Another aspect that was covered in multiple reviews was the use and availability of public datasets, which is paramount to expand the COVID-19 research capabilities.

Model generalization has also been tackled in numerous studies as it is an important aspect to be considered while building deep learning-based models. While the reviews have covered the majority of the research taking place and the challenges accompanied by them, only Shorten et al. [52] accounted for extending work via privacy-preserving methods and mentioned research taking place through other deep learning paradigms such as meta-learning [126] and self-supervised learning [127]. Apart from these, the readmission risk of COVID-19-recovered patients can also be analyzed using a predictive model. Many ML- and DL-based predictive models have been designed to predict the readmission risk of patients discharged from hospitals for various diseases [128, 129]. Increased readmission rates may be liable to high healthcare cost and risk of inpatient hospital mortalities. Several works have been carried out to improve the performance of these predictive models using evaluation metrics [130, 131]. Similarly, many studies have been conducted regarding the COVID-19 case readmission rates and factors [132, 133].

In the field of medicine, data privacy is of utmost importance and is always the leading cause for the shortage of open-source data. Addressing this issue should be the first among the list of challenges concerning COVID-19. One of the main reasons for having such expansive development and testing is because of the large amounts of open-source data present (including open accessing all research), which is generally absent for other diseases. Self-supervised learning approaches have proven to surpass the usual supervised deep learning methods in [134, 135] and should be given more importance and consideration when topics of extension and challenges are brought upon. There is also a major gap in accounting for the research conducted in terms of prognosis for COVID-19. There is no single review that focuses on this aspect. In terms of medical image analysis, few solutions are addressed to the challenges mentioned in [52]. To the best of our knowledge, the previous reviews missed to cover the topics discussed above. Additional information is all part of recent developments, which have taken place post the drafting of those reviews.

### 3.1. Extension of Discussion on the Limitations of Deep Learning Approaches Discussed in Shorten et al. (2020) [52]

(a) *Explainability*: deep learning models are often called black box models due to their non-interpretive behavior. This highly disregards using deep learning models on sensitive real-world tasks such as medical image analysis and has hence turned into a nontrivial issue. With the focus here being the same, there are ample explainable techniques that have come up to aid in explaining vision-based deep learning models.  Table 7 shows the current state-of-the-art methods used to help interpret vision-based deep learning models. Score-CAM eliminates the dependence on gradients (as seen in Grad-CAM) by securing the weight of individual activation maps, by virtue of its forward passing score on the aimed target class, which results in a linear combination of the activation maps and weights. EVET [135] proposes a heuristic pipeline for strengthening the visual explanations by applying image transformations. Explainability in segmentation tasks (primarily done by U-Nets) is a field that is still being heavily explored. Initial attempts have been done by adapting Grad-CAM to segmentation in the form of SEG-GRAD-CAM [136]. The origin of the above work comes from [137]. Explainable models can benefit the medical image analysis pipeline in many ways. It helps understand where the model is focusing on the image, increase user confidence, and inspect the model at a deeper level, which in turn helps in debugging the model as well.
(b) *Generalization Metrics*: precision is generally the major metric taken into consideration while accounting for a fair metric for medical image classification methods. While considering segmentation, the authors in [138] give a detailed description regarding which metrics to consider. They also mention the use of precision here as well. A detailed study on generalization concepts and metrics can also be studied in [139].
(c) *Learning From Limited Labeled Datasets or Unlabeled Data:* primary focus on two paradigms of learning is as follows:
  - Meta-Learning: it follows the approach of learning to learn. It is used to adapt to learn new environments and in a quicker fashion greatly aligns with the demand of COVID-19 research. It also requires lesser data samples. In [118], a trainable n-shot deep meta-learning framework was built to classify COVID-19 cases with limited training CXR images. Another aspect of meta-learning is neural architecture search (NAS) and that has been observed to work better than many baseline models [140].
  - Self-Supervised Learning: it is a subgroup of unsupervised learning, which works on the basis of training the deep learning model explicitly with automatically generated labels. As Figure 10 depicts, the process involves learning visual features from pretext task (tasks predesigned for networks to deal with) and acts as a pre-trained model for other downstream tasks (computer vision applications to examine the self-supervised learned feature quality) via fine-tuning. References [133, 134] have rivaled the top-performing models in image tasks, even surpassing the supervised methods. Reference [141] showed that the combination of data augmentation and self-supervised learning has outperformed all previous approaches in severity assessment.
(d) *Data Privacy*: a detailed discussion of data privacy is given in [52]. To extend on the avenues mentioned there, the use of differentially private federated neural architecture search [142] is recommended to preserve data privacy. Through this method, a model can be tested on several subsets of data, which contain varied distributions and distinctions from other datasets and in parallel keep any information about the various data samples completely privatized. Although the method is very computationally demanding, it can help screen through different samples of data and greatly test the robustness of any model.  Figure 11 depicts the working of both NAS and federated NAS (FNAS) [143]. An application of federated learning in terms of prognosis can be seen in [144]. A noise implementation algorithm is integrated with a cross-device federated learning, such that the initial symptom prognosis can be achieved during a pandemic like COVID-19.

## 4. Pre- and Post-Processing Techniques for COVID-19 Medical Image Analysis

### 4.1. Preprocessing

Preprocessing is a crucial part of vision models' pipeline. The process involves performing operations at the lowest level of abstraction. The objective is to enhance the picture information that suppresses undesired deformities or improves the image features necessary for continued transformations, which is mainly linked with generating higher accuracy in models. Even simple techniques such as resizing or cropping the image can make major difference in deep learning models. For example, cropping out the redundant parts of a scan can help the deep learning model avoid unnecessarily parsing through that spatial information to concentrate on the more essential areas of the scan. Certain models require specific size of input images to fit in. In such situations, rescaling the image is completely unavoidable.

Figure 12 depicts a chest CT scan being put through contrast-limited adaptive histogram equalization (CLAHE) in comparison with an original CT image. A clear depiction of sharper visual features after CLAHE is applied, which makes it easier for the model to develop and correlate these visual cues.  Figure 13 illustrates how the preprocessing step can also help better express the image features through image enlargement. The enlarged points are first targeted (shown as question marks) and then filled through interpolation. A comparative image is also shown with no interpolation done. In addition to the techniques mentioned in Table 8, there are certain methods that can aid in preprocessing. Data augmentation is a widely used method in much literature to help increase the training sample size. GANs have also been applied to increase the sample size [153]. Noise removal techniques without losing the significant edges can also be used to enhance the images [154].

### 4.2. Post-Processing

Post-processing generally directs to improvement in the images after the model has given an output, but in the case of medical image analysis, it mainly involves generating inferences from the model outputs via explainability measures. The basis of most techniques is class activation maps [137]. These methods are used to pinpoint the focus of the model and understand whether the output generated is on the basis of the detection of the actual disease and not any other factors. The extensions made to [137] are discussed in Section 3.1.1. In [155], a method called the Peekaboo training scheme was used, in which a two-stage patch crop-and-drop strategy promotes the model to furnish activation maps for every target concept.

## 5. Discussion

In this section, we discuss additional challenges faced while conducting experiments and how the work done with respect to COVID-19 can help the field of medical image analysis in general.

### 5.1. Challenges Faced

Reviewing of multiple literature samples led to the identification of multiple challenges present in the domain, a few of which are already covered in Section 3.1. In this section, another set of challenges that have been discovered is elucidated.

- Interclass analogy and intraclass deviation of pneumonia lesions: COVID-19 pneumonia, which is also caused by viral infection, contains indicative overlay of features and radiological image characteristics with other viral pneumonia leading to the interclass analogical problem. Another problem that arises while dealing with the pulmonary medical images is the intensity in-homogeneity problem caused by the closeness of gray level between the different soft tissues, resulting in segmentation and detection difficulties [156]. Detecting the anomalous features from the medical images becomes challenging due to the noise impedances from the tissues and lesions. The infected region may still contain some non-lesion regions with wide variations in tissues, which further makes it complicated to differentiate.
- Generalization and reproducibility: the COVID-19 detection algorithms proposed by various researchers produce great results for the particular small dataset used in that work. When these trained classifier algorithms are implemented on larger unseen data, they may not be able to generalize their performance. Moreover, problems arise in reproducing the similar performance on other multicenter datasets. One such solution to this problem is the use of vision transformers, which have demonstrated superior performance and greater generalization prowess. These are of paramount importance in the context of a deployment scenario [157].
- Data source learning problem of ML and DL: on applying neural network-based COVID-19 detection protocols to multicenter datasets, most of the detection systems tend to learn the source of dataset, their imaging protocols, mode, and so on, rather than learning the discriminative features among the various classes. Such kind of algorithms may not be fair enough when generalized for different data [158].
- Spread and contamination: contamination of the scanners is also an issue that needs to be considered. There is a great possibility of disease spread during scanning; hence, the radiologists must assure that the scanners are maintained clean after every scanning process.

### 5.2. Future Scope: Utilizing COVID-19 Medical Image Analysis Research in Other Fields

As seen, enormous amounts of effort take place to furnish new methods through deep learning strategy to tackle the problems of COVID-19 detection. A few potential avenues have been mentioned in this section, which can in general help to extend the field of medical image analysis.

- Medical model weights and baseline architectures: utilizing model weights built upon disease-affected scans has shown to improve the efficiency in models [87]. Particular to COVID-19, CheXNet [159] weights utilized in models instead of the usual ImageNet weights have been shown to increase the model [160], which can be utilized to detect other diseases as well. General vision problems are quite different when compared to dealing with medical images such as MRIs, CTs, and PET scans. Training models that are based on the weights gained from training on such images should furnish more accurate models. Apart from COVID-19, there are many other diseases that can be detected from radiographs. As DenseNet is seen to do well for COVID-19 (both from pre-training and for customized models), it should be fair enough for other diseases as well and can act as a good starting point for future researchers to expand existing works.
- Expanding the community and model testing: there are many introductory materials focused on COVID-19 and medical image analysis. This can help build the community further and attract novices to the field. Testing models on scarce datasets make it quite difficult to generate inference about the model's performance. With the massive open-source data available, it also allows potential researchers to realistically test their models and architectures. The variety of data present also helps in testing the model for generalizability, which is one of the biggest obstacles to surmount while utilizing deep learning-based methodologies.

## 6. Conclusion

A comprehensive description on the various COVID-19 detection techniques using medical image analysis has been described in this study. The cause, effect, challenges, limitations, and other retrospective discussions on COVID-19 medical image analysis have been discussed through this study to best feature the importance of carrying out more research on this area to reduce the increased mortality count faced by the world. DL can improve the disease diagnosis efficiency by precisely locating the infections in the medical images in a faster and accurate manner. The preceding COVID-19 analysis methodologies proposed by various researchers can be used only as a reinforcement technique to assist the medical teams in highly populated areas and in situations requiring quicker diagnosis. The problems such as unavailability of enough and accurate labeled data, generalization and reproducibility of preceding algorithms for multicenter large datasets, and difficulty to isolate COVID-19 against other pneumonia cases due to the closeness of gray level of the soft lung tissues have been highly challenging to design a diagnostic system with high reliability and accuracy. An intelligent and accurate computer-assisted COVID-19 diagnostic system employing adaptive deep learning models with active/incremental learning is the need of the hour to combat the evolving coronavirus.

## Figures and Tables

**Figure 1:** (a) Radiological image acquisition (courtesy: newsnetwork.mayoclinic.org/discussion/mayo-clinic-radio-lung-cancer-updatehousehold-health-hazardsprediabetes). (b) (A) Axial chest CT image (non-enhanced) of a positive RT-PCR-confirmed 70-year-old man showing ground-glass opacities along with dilated segmental and subsegmental vessels prominent on the right side. (b) (B) CXR showing pulmonary hypertension, mitral insufficiency, and atrial fibrillation along with COVID-19 contagion in an 83-year-old man (arrows indicating ground-glass opacity findings in the upper right lobe and consolidation findings in the lower left lobe of the lungs) (arrows) (courtesy: radiologyassistant.nl).

**Figure 2:** Example of DenseNet architecture.

**Figure 3:** 2D feature extraction by filters and kernels from images through convolution operations.

**Figure 4:** COVID-19 detection system.

**Figure 5:** Flow of review on different medical imaging analysis tasks.

**Figure 6:** Sample residual connection used in ResNet [40].

**Figure 7:** Sample U-Net architecture for medical image segmentation. ^*∗*^ in the legend indicates that the filter is followed by a batch normalization layer and a ReLU function.

**Figure 8:** Inferences from the review of COVID-19 medical image analysis.

**Figure 9:** Generalized pipeline of COVID-19 detection from radiological image modalities.

**Figure 10:** General self-supervised learning pipeline. PTT: pretext task training; DTT: downstream task training.

**Figure 11:** General federated learning pipeline.

**Figure 12:** Original CT image versus CLAHE-processed CT image [145].

**Figure 13:** Depiction of a pipeline for enlarging an image through interpolation.

**Table 1:** Machine learning techniques tried and true in preceding COVID-19 medical image analysis.

Algorithm	Summary
RF^1^ [17]	Utilized quantitative features of CT scans
SVM [18]	Tested SVM (RBF)^1^ on raw and modified CT images
KNN [18]	Tested KNN (*N* = 21)^1^ on raw and modified CT images

^1^RF indicates random forest algorithm. RBF indicates radial basis function. *N* indicates the number of neighbors considered. Rest all were set to the general settings.

**Table 2:** Evolution of CNNs since 1959. The table describes primary points of novelty that motivated new architectures to be produced.

Architecture	Primary focus and novelty	Author and year
Simple and complex cells [28]	Described cells in the human cortex.	Hubel & Wiesel (1959)
	Proposed its use case in pattern recognition.	
Neocognitron [29]	Converted the cell idea from [28] into a computational model.	Fukushima (1980)
LeNet-5 [30]	First modern CNN.	Lecun et al. (1998)
	Composed of two convolution layers with three fully connected layers. Introduced the MNIST database.	
AlexNet [31]	Implemented overlapping pooling and ReLU [32].	Krizhevsky et al. (2012)
	Non-saturating neurons are used.	
	Facilities' effective usage of GPU-driven methods.	
VGG-16 [33]	Made an exhaustive evaluation on architectures of increasing depth.	Simonyan and Zisserman (2014)
	Used architectures with tiny (3 × 3) convolution filters.	
Inception [34]	Dimensions of network are increased while keeping the computational budget constant.	Szegedy et al. (2015)
	Utilized the Hebbian principle and multiscale processing.	
Modified VGG-16 [35]	Proposed that if a model is strong enough to fit a large dataset, it can also fit to a small one.	Liu and Deng (2015)
ResNet [36]	Presented a residual learning framework.	He et al. (2015)
	Allowed building larger models with deeper layers through skip connections. Paved the way for more variants [37, 38].	
Xception [39]	Presented a depth-wise separable convolution as an inception module with a maximally large number of towers.	Chollet (2016)
MobileNets [40]	Made for mobile and embedded vision applications.	Howard et al. (2017)
	Streamlined architecture using depth-wise separable convolutions.	
ResNeXt [41]	Presented cardinality (size of the transformation set) as a key factor along with the dimensions of an architecture.	Xie et al. (2017)
DenseNet [42]	Complete intra-layer connections among all singular connections in a feed-forward fashion.	Blei et al. (2017)
	Strengthens feature propagation and encourages feature reuse.	
Squeeze-and-excitation block [43]	Adaptively recalibrates channel-wise feature responses by explicitly modelling interdependencies between channels.	Hu et al. (2018)
Residual inception [44]	Combined residual and inception module.	Zhang et al. (2018)
NASNet search space [45]	Designed a new search space to enable transferability.	Zoph et al. (2018)
	Presented a new regularization technique—scheduled drop path	
EfficientNet [46]	Proposed a novel scaling technique that scales all the dimensions (width/resolution/depth) uniformly using a compound coefficient.	Tan and Le (2019)
Normalizer-free models [47]	Developed an adaptive gradient clipping technique to overcome instability.	Brock et al. (2021)
	Designed a significantly improved class.	

**Table 3:** A summary of research reviewed on COVID-19/non-COVID-19 pneumonia diagnosis.

Work	Image modality	Dataset size	Method used	Accuracy (in %)	Sensitivity or recall (in %)	Specificity (in %)	AUC (in %)	Precision (in %)	F1 score
Harmon et al. [54]	CT	(i) 1029 COVID-19	DenseNet-121 and AH-Net segmentation	90.8	84	93	94.9	NA	NA
		(ii) 1695 non-COVID-19							
		Pneumonia							

Ouyang et al. [55]	CT	(i) 3389 COVID-19	Dual sampling	87.5	86.9	90.1	94.4	NA	0.82
		(ii) 1593 CAP	Attention network with ResNet-34						

Wu et al. [56]	CT	(i) 331 COVID-19	Multiview fusion model using ResNet-50	76	81.1	61.5	81.9	NA	NA
		(ii) 114 other pneumonia							

Ardakani et al. [57]	CT	(i) 510 COVID-19	ResNet-101	99.51	**100**	99.02	**99.4**	NA	NA
		(ii) 510 non-COVID-19							

Sun et al. [58]	CT	(i) 1495 COVID-19	Adaptive feature	91.79	93.05	89.95	96.35	NA	NA
		(ii) 1027 CAP	Selection-guided deep forest—SVM						

Narin et al. [59]	CXR	(i) 341 COVID-19	ResNet-50	99.5	99.4	99.5	NA	98	**0.987**
		(ii) 1493 viral pneumonia							
		(iii) 341 COVID-19		**99.7**	98.8	**99.8**	NA	98.3	0.985
		(iv) 2772 bacterial pneumonia							

Zhang et al. [63]	CXR	(i) 100 COVID-19	Residual CNN with anomaly detection head	NA	96	70.65	95.18	NA	NA
		(ii) 1431 pneumonia							

Abraham and Nair [64]	CXR	(i) 453 COVID-19	Combination of multi-CNN	91.16	98.5	NA	96.3	85.3	0.914
		(ii) 497 non-COVID-19							
		Pneumonia							
		(i) 71 COVID-19		91.44	98.6	NA	91.1	**98.6**	0.986
		(ii) 7 non-COVID-19							
		Pneumonia							

Autee et al. [67]	CXR	(i) 868 COVID-19	StackNet-DenVIS	95.07	99.40	94.61	98.40	NA	NA
		(ii) 9085 non-COVID-19							

Bold values represent the best result obtained for each performance metric among all the methodologies compared.

**Table 4:** A summary of research reviewed on COVID-19/non-COVID-19 pneumonia/normal or non-pneumonia diagnosis.

Work	Image modality	Dataset size	Method used	Accuracy (in %)	Sensitivity or recall (in %)	Specificity (in %)	AUC (in %)	Precision (in %)	F1 score
Li et al. [70]	CT	(i) 1292 COVID-19	COVNet	NA	90	96	96	NA	NA
		(ii) 16325 non-COVID-19 pneumonia							
		(iii) 1735 CAP							

Wang et al. [71]	CT	(i) 1315 COVID-19	Prior-attention	93.3	87.6	95.5	NA	NA	NA
		(ii) 963 normal	Residual model 3D ResNets						
		(iii) 2406 ILD							

Hasan et al. [72]	CT	(i) 118 COVID-19	LSTM using Q-deformed entropy and deep features	**99.68**	NA	NA	NA	NA	NA
		(ii) 96 pneumonia							
		(iii) 107 normal							

Butt et al. [73]	CT	(i) 219 COVID-19	3D ResNets with location attention mechanism	86.7	98.2	92.2	**99.6**	81.3	0.839
		(ii) 224 IAVP							
		(iii) 175 normal							

Song et al. [74]	CT	(i) 777 COVID-19	DRENet	93	93	NA	NA	93	0.93
		(ii) 505 bacterial pneumonia							
		(iii) 708 normal							

Toğaçar et al. [75]	CXR	(i) 371 COVID-19	SVM—social	99.27	98.33	99.69	NA	98.89	0.9858
		(ii) 98 pneumonia	Mimic optimized deep features						
		(iii) 65 normal							

Wang et al. [68]	CXR	(i) 358 COVID-19	COVID-Net	93.3	91	NA	NA	NA	NA
		(ii) 5538 non-COVID-19 pneumonia							
		(iii) 8066 normal							

Nishio et al. [80]	CXR	(i) 215 COVID-19	VGG-16 with conventional and mix-up augmentation	83.7	90.9	NA	NA	NA	NA
		(ii) 533 non-COVID-19 pneumonia							
		(iii) 500 normal							

Canayaz [81]	CXR	(i) 364 COVID-19	MH-Net	99.38	**99.39**	**99.69**	NA	**99.39**	**0.9938**
		(ii) 364 pneumonia							
		(iii) 364 normal							

Almalki et al. [82]	CXR	(i) 284 COVID-19	CoVIRNet feature extractor with RF	97.29	97.02	NA	NA	97.74	0.9732
		(ii) 327 viral pneumonia							
		(iii) 330 bacterial pneumonia							
		(iv) 504 normal							

Bold values represent the best result obtained for each performance metric among all the methodologies compared.

**Table 5:** Performance metrics used in COVID-19 detection.

Performance metric	Accuracy	Sensitivity/recall	Specificity	Precision	F1 score
Formula	(TP+TN)/(TP+FP+TN+FN)	TP/(FN+TP)	TN/(FP+TN)	TP/(FP+TP)	(2*∗*(*R∗P*))/(*R*+*P*)

TP—true positive, TN—true negative, FP—false positive, FN—false negative, *R*—recall, and P—precision.

**Table 6:** Merits and limitations of existing review papers exploring the broad depth of COVID-19 research in terms of medical imaging, medical image analysis, machine learning, and deep learning.

Review paper	Merits	Limitations
Ozsahin et al. [119]	Classified different groups of studies.	Only highlights result and techniques without any intuition as to why either are used.
	Added a severity constraint.	Includes segmentation models within classification studies.
Shoeibi et al. [120]	Includes a forecasting study of coronavirus prevalence in multiple countries.	Certain figures depict subpar comparisons and include unnecessary comparison samples.
	Includes pre- and post-processing techniques used in various COVID-19 detection approaches.	The review is more focused on architectures utilized rather than the inference generated from the literature.
Pham [97]	Presents many strong inferences on pre-trained networks.	Should have considered the use of the Matthews correlation coefficient (MCC) [121] as binary classification was considered.
	Alleviates the task of data augmentation. Empirically proved DenseNet-201 works best.	
Shorten et al. [52]	Pinpoints key discussions in regards to deep learning approaches and the challenges faced by same in multiple domains apart from medical imaging.	Falsely claims the first paper to review in a deep learning point of view for COVID-19 analysis.
	Explores several supporting domains such as federated learning, meta-learning, and self-supervised learning, which is missed in most reviews.	Compares paper to other “artificial intelligence”-based methods to their approach.
Alsharif et al. [122]	Attempts to compare deep learning to machine learning approaches.	Fails to dive deep into the problem and hence causes incorrect generalization of methods.
Joy et al. [123]	The review is inclined to help beginners in the field.	No challenges are mentioned or analyzed.
	It poses an extensive study covering various approaches and architectures.	
Alghamdi et al. [124]	Gives in-depth analysis about architectures and the various constraints in tandem to them such as data, explainability, and more.	Does not consider the SOTA methods in explainability terms.
		Fails to address other possible learning paradigms and privacy-preserving methods.
		Should be mentioned as the review is architecture-dominated.
Islam et al. [125]	Gives an extensive study on open challenges.	Limitations are covered in the paper.
	Highlights the data partitioning techniques.	

^1^While there are other reviews present, they were either extremely short, or did not contain valuable information, or were mostly covered in the mentioned reviews.

**Table 7:** State-of-the-art explainable techniques for vision-based deep learning models.

Task	Explainable method
Classification	Grad-CAM [48]
	Score-CAM [49]
	EVET [135]
Segmentation	SEG-GRAD-CAM [136]

**Table 8:** List of preprocessing techniques used for analyzing radiological images.

Reference	Technique	Utilization
Pizer et al. [146]	Adaptive histogram equalization	Improves contrasts in images.
Veldhuizen and Jernigan [147]	Wiener filter	Produces an estimate of a desired or target random process.
Lehmann et al. [148]	Interpolation	Best estimation of a pixel's color and intensity in context to the values at neighboring pixels.
Tian et al. [149]	Binarization	Transforms data features of any entity into vectors of binary numbers.
Yadav et al. [145]	CLAHE	Amplifies the contrasts.
		Works on small regions called tiles.
Prabha and Kumar [150]	Smoothing filter	Utilized in blurring regions.
Kociołek et al. [151]	Normalization	Changes the range of pixel intensity values.
Gungor [152]	Wavelet transform	Reduces noise in images.
		Decomposes special patterns hidden in mass of data.

## Data Availability

The data supporting this systematic review are from previously reported studies and datasets, which have been cited.
